This article has been retracted.

# Task-Oriented Intelligent Solution to Measure Parkinson's Disease Tremor Severity

**DOI:** 10.1155/2021/9624386

**Published:** 2021-09-10

**Authors:** Ghayth AlMahadin, Ahmad Lotfi, Marie Mc Carthy, Philip Breedon

**Affiliations:** ^1^School of Science and Technology, Nottingham Trent University, Clifton Lane, Nottingham NG11 8NS, UK; ^2^ICON PLC, South County Business Park, Dublin 18, Ireland

## Abstract

Tremor is a common symptom of Parkinson's disease (PD). Currently, tremor is evaluated clinically based on MDS-UPDRS Rating Scale, which is inaccurate, subjective, and unreliable. Precise assessment of tremor severity is the key to effective treatment to alleviate the symptom. Therefore, several objective methods have been proposed for measuring and quantifying PD tremor from data collected while patients performing scripted and unscripted tasks. However, up to now, the literature appears to focus on suggesting tremor severity classification methods without discrimination tasks effect on classification and tremor severity measurement. In this study, a novel approach to identify a recommended system is used to measure tremor severity, including the influence of tasks performed during data collection on classification performance. The recommended system comprises recommended tasks, classifier, classifier hyperparameters, and resampling technique. The proposed approach is based on the above-average rule of five advanced metrics results of four subdatasets, six resampling techniques, six classifiers besides signal processing, and features extraction techniques. The results of this study indicate that tasks that do not involve direct wrist movements are better than tasks that involve direct wrist movements for tremor severity measurements. Furthermore, resampling techniques improve classification performance significantly. The findings of this study suggest that a recommended system consists of support vector machine (SVM) classifier combined with BorderlineSMOTE oversampling technique and data collection while performing set of recommended tasks, which are sitting, stairs up and down, walking straight, walking while counting, and standing.

## 1. Introduction

Parkinson's disease (PD) is one of the most widespread neurodegenerative disorders affecting more than 10 million globally. The four main motor symptoms of PD are tremor (rhythmic shaking movement), bradykinesia (slowness of movement), rigidity (muscle stiffness), and postural instability (impaired balance) [1]. Tremor defines one-sided, involuntary, rhythmic motions in the limbs, often in the hands. PD tremors can be divided into three types: rest tremor (RT), kinetic tremor (KT), and postural tremor (PT) [2]. The RT takes place at 4–6 Hz in a relaxed and supported limb of 70%–90% of PD patients. The PT arises when a person performs an antigravity position, such as extending arms at a frequency between 6 and 9 Hz. The PT occurs when a person maintains a position against gravity, such as stretching arms at a frequency between 6 and 9 Hz. The KT is a form of tremor that happens at a frequency between 9 and 12 Hz during voluntary gestures such as drawing, writing, or touching of the tip of the nose [2].

Currently, Parkinson's tremor severity is scored based on the Movement Disorders Society's Unified Parkinson's Disease Rating Scale (MDS-UPDRS) from 0 to 4 with 0, normal; 1, slight; 2, mild; 3, moderate; and 4, severe [3]. However, The MDS-UPDRS is a subjective assessment that mainly relies on visual observations and on the clinicians' skills and experience [4]. There is evidence showing that the MDS-UPDRS has high inter- and intrarater variability [5]. Thus, a patient's tremor could be given a score by one clinician and, at the next visit, evaluated by another clinician and assigned a higher score. In this case, it is difficult to interpret these two different scores, whether symptoms worsen or are due to subjectivity. In addition, the assessment often takes time and involves advanced official training to improve the coherence of data acquisition and interpretation [6].

Advances in sensing technologies combined with artificial intelligence (AI), specifically machine learning (ML) techniques, have enabled the development of new approaches for objective assessment of PD motor symptoms [7]. These approaches basically consist of four main steps: data collection, signal processing, features extraction, and classification algorithms. The data collection can be classified according to performed tasks into two main groups: scripted tasks and unscripted tasks [8]. Scripted motor tasks (predefined motor tasks) are performed under supervision in laboratory settings (e.g., Part III of MDS-UPDRS, motor examination, structured Activities of Daily Living (ADL) tasks), while unscripted tasks are ADL performed under free-living conditions without any supervision or instruction.

Several objective methods have been proposed for measuring and quantifying PD tremor from data collected during performing scripted and unscripted tasks [9]. For example, Giuffrida et al. [10] used Kinesia™  system (https://glneurotech.com/kinesia/), which is a sensor that integrates accelerometer and gyroscope, for PD tremor severity score assessment. In this study, the data were collected from Kinesia™ system placed on the middle finger of the most affected hand, while the subjects were performing three scripted tasks from Unified Parkinson's Disease Rating Scale (UPDRS), including rest, postural, and kinetic tremor. This study utilised a multiple linear regression algorithm with coefficient of determination, *r*2 for evaluation, and achieved *r*2=0.89 for rest tremor, *r*2=0.90 for postural tremor, and *r*2=0.69 for kinetic tremor. Similarly, Niazmand et al. [11] have used data collected from integrated pullover triaxial accelerometers, while subjects performed rest and posture UPDRS motor tasks. The correlation between the measurements from accelerometers and UPDRS scores calculated and achieved 71% sensitivity of detecting tremor and 89% sensitivity of detecting posture tremor.

Rigas et al. [12] conducted a study to estimate tremor severity using a set of wearable accelerometers, while subjects were performing ADL tasks. A Hidden Markov Model (HMM) was employed to estimate tremor severity. They have achieved 87% overall accuracy with 91% sensitivity and 94% specificity for tremor 0, 87% sensitivity 82% specificity for tremor 1, 69% sensitivity and 79% specificity for tremor 2, and 91% sensitivity and 83% specificity for tremor 3.

Authors in [13] collected triaxial accelerometer data from PD patients using a smartwatch, while they are performing five motor tasks including sitting quietly, folding towels, drawing, hand rotation, and walking. They have used support vector machine (SVM) to predict tremor severity into three tremor levels, 0, 1 and 2, where 2 represents tremor severities 2, 3, and 4. The model achieved 78.91% overall accuracy, 67% average precision, and 79% average recall.

A common limitation in most of the previous studies was that the authors did not take into consideration data collection influence on tremor measurement. Moreover, previous studies did not report advanced performance metrics such as sensitivity, specificity, F-score, Area Under the Curve (AUC), and Index of Balanced Accuracy (IBA), which are very important to evaluate classification models, particularly in medicine field where misclassification can lead to unnecessary treatment. In addition, most of the previous studies did not take into consideration imbalanced classes distribution among collected data.

An extensive review of the literature showed that only few studies have explored different aspects of tremor measurement. For example, in [14], the authors explored two tasks (standing, sitting) effects on tremor measurement and the correlation with clinical score were 0.70 in case of standing and 0.75 in case of sitting. In [15], authors reported tremor measurement of the left and the right hands and the correlation were 0.88 and 0.77, respectively. In [16], the tremor severity was quantified under two conditions, while patients were on medication and off medication and showed that the correlation with clinical score is higher when patients were on medication (0.779), while it was 0.638 when patients were off medication. This indicates a need to explore different aspects of tremor measurement that might improve the objective evaluation PD tremor.

The research to date has tended to focus on proposing a tremor severity classification approach without discrimination tasks effect on classification and tremor severity detection, even though motor examination of PD is a key aspect of tremor assessment [3]. Therefore, in order to propose a recommended system to measure tremor, it is essential to suggest and validate a method that includes a protocol of data collection including tasks where the tremor severity is highly distinguishable besides signal processing, features extraction, and classification algorithms. In addition, it is important to take into consideration a well-known challenge in ML algorithms development in medical applications, which is the issue of imbalanced classes distributions or the inadequacy of a class or some classes in the data, which cause a missclassification that can lead to wrong assessment [17]. Therefore, several methods have been suggested to address the imbalanced data issue [18], and one of these methods is the resampling techniques, which have been shown to be an excellent solution for handling imbalanced data in various applications [19].

This study presents a novel comprehensive method to develop and validate a recommended system to measure and quantify PD tremor severity, including recommended tasks for data collection from different sensors, signal processing, robust features extraction, exploring various classifiers with exhaustive hyperparameters tuning with, and without resampling techniques. The development was validated through different metrics such as accuracy, F1-score, geometric mean (G-mean), Index of Balanced Accuracy (IBA), and Area under the Curve (AUC).

## 2. Materials and Methods

To define a recommended system for PD tremor measurement, three main components should be identified, best task, best classifier, and best resampling technique.  Figure 1 illustrates the proposed framework to find the recommended system(s) to detect tremor severity from four different subdatasets.

Four subdatasets were prepossessed independently in the first phase to eliminate reliance on sensor orientation and nontremor data and artefacts. Various time and frequency domains features were extracted from the prepossessed data in the second phase. In the third phase, data was split into training, evaluation, and test subsets. A copy of training data was resampled by six different resampling techniques independently, in the fourth phase. In the fifth phase, two copies of the training data (with resampling and without resampling), and the test data were applied to six different classifiers. The classification results were evaluated by five metrics in the sixth phase. In the seventh phase, the results passed to recommended tasks framework, recommended classifier, and resampling techniques framework. Each step is described in detail in the subsequent sections.

The training data 60%, test data 25%, and evaluation data 15% were selected randomly from entire dataset and does not belong to specific patients; in other words, the splitting were based on tremor severity of each segmented window. The training and test data were used to evaluate and to identify best classifier and resampling techniques combination (potential recommended systems), while the evaluation data were used to evaluate the identified potential recommended systems as an external dataset.

### 2.1. Dataset

Tremor dataset (it is available at https://www.michaeljfox.org/news/levodopa-response-study) was taken from Levodopa response trial wearable data from the Michael J. Fox Foundation for Parkinson's research (MJFF) [20]. The data were collected from 30 PD patients over four days from wearable sensors in both laboratory and home environments using different devices: a Pebble Smartwatch (https://www.fitbit.com/pebble), GENEActiv accelerometer (https://www.activinsights.com/products/geneactiv/), and a Samsung Galaxy Mini smartphone accelerometer. On the first day of data collection, participants came to the laboratory on their regular medication regimen (on medication) and performed set ADL tasks and tasks of motor examination of the MDS-UPDRS [3], which is used to assess motor symptoms. On the second and third days, accelerometers data were collected while participants were at home and performing their usual activities. On the fourth day, the same procedures that were performed on the first day were performed once again, but the participants were off medication for twelve hours. For each task, on the first and the fourth days, symptom severity scores (rated 0-4) were provided by a clinician.

The list of tasks performed can be categorised into two groups. The first group includes tasks which involve direct wrist movement, that is, drawing on a paper, writing on a paper, taking a glass of water and drinking, folding a towel, finger to the nose (left and right arms), assembling nuts and bolts, organising sheets in a folder, repeated arm movement (left and right arms), and typing on a computer keyboard. The second group includes tasks that do not involve direct wrist movement which are sitting, standing, walking downstairs, walking upstairs, sit to stand, walking while counting, walking through a narrow passage, and walking straight. In this study, only labelled data was used, which is the data collected on day one and day four from GENEActiv accelerometer and Pebble Smartwatch as shown in Figure 2.

Table 1 shows classes (severities) distribution of 103080 instances (windows) segmented from collected data. It is clear how data distribution is skewed towards less severe tremor, and this bias can cause significant changes in classification output. In this situation, the classifier is more sensitive to identifying the majority classes but less sensitive to identifying the minority classes.

### 2.2. Signal Processing

In order to avoid dependency on sensor orientation and processing signal in three dimensions, the first step in this phase is to calculate the vector magnitude of three orthogonal acceleration, namely, *A*_*X*_, *A*_*Y*_, and *A*_*Z*_. To keep tremors bands and to eliminate low and high-frequency bands, as suggested by earlier work [2], a band-pass Butterworth filters with cut-off frequencies 3 − 6 Hz for RT and 6 − 9 Hz for PT and 9 − 12 Hz for KT are applied in the second step. The filtered signals were segmented using sliding windows of four seconds length with 50% overlap.

### 2.3. Features Extraction

Different features in time and frequency domains were extracted from three frequency bands, 3 − 6 Hz for RT, 6 − 9 Hz for PT, and 9 − 12 Hz for KT, to form a 102 features vector. Frequency domain features were extracted after transforming the signal to frequency domain using Fast Fourier Transform (FFT) according to the following equation:

(1) $$\begin{array}{c} F\left(k\right)=\sum_{t=0}^{W_{l}-1}a_{t}e^{\left(-j2\pi kt/W_{l}\right)},\;\text{for }k=0,\ldots ,W_{l}-1, \end{array}$$

where *F*(*k*) complex sequence that has the same dimensions as the input sequence (*a*_*t*_)_*t*=0_^*w*_*l*_^ and *e*^−*j*2*π*/*W*^ is a primitive *N*^th^ root of unity.

The extracted features have been specifically chosen to discriminate tremor severity such as central tendency, dissimilarity, distribution, autocorrelation, dispersion, data shape, stationarity, and entropy. Previous research has established that features such as mean, max, energy, number of peaks, and number of values above and below mean and median are highly correlated with tremor severity [21, 22]. Likewise, tremor severity is highly correlated with signal amplitude [23], as high signal amplitude indicates high tremor MDS-UPDRS score and vice versa.

The standard deviation has been chosen to measure signal dispersion as an appropriate way to quantify tremor severity [24]. Skewness and kurtosis have been selected to measure data distribution because tremor signals have higher kurtosis values than nontremor signals [25], while nontremor signals have higher skewness values than tremor signals [21].

A prior study has shown that tremor intensity defines the severity of tremor [2], and since tremor severity correlated with frequency subbands or bandwidth spread [11], the Power Spectral Density (PSD) can be used to quantify tremor intensity at different frequencies. Thus, three features have been calculated: fundamental frequency, median frequency, and frequency dispersion. The fundamental frequency, which is the frequency, has the highest power of all the frequencies in the spectrum. The median frequency, which is the frequency, splits the PSD into two equal parts. Frequency dispersion is the width of the frequency band that comprises 68% of the PSD. The difference between the fundamental frequency and the median frequency was taken from previous work as an additional feature since the fundamental frequency of tremors could vary between PD patients [26]. Spectral centroid amplitude (SCA), which is the weighted power distribution, and maximum weighted Power Spectral Density (PSD) have been selected to measure spectral energy distribution [27].

The PD tremor is a rhythmic motion, hence autocorrelation and sample entropy features that could measure regularity and complexity in time series data, where tremor motions' autocorrelation and sample entropy are considerably less than nontremor motions that has been demonstrated by earlier work [28, 29]. The complexity-invariant distance (CID) [30], the sum of absolute differences (SAD) [15], and another complexity features have been used to identify tremor. SAD and CID measures time series complexity based on peaks and valleys, as the more complex signal has more peaks and valleys. Consequently, the tremor signal is more complex because tremor frequency and amplitude are higher than nontremor signal; in other words, the tremor signal has a higher number of peaks and valleys. A list of the extracted features and their descriptions is presented in Table2.

## 3. Resampling Techniques

This section presents a brief about resampling techniques employed in this study. Resampling methods can be categorised into three groups: oversampling, undersampling, and hybrid (combination of over- and undersampling).

### 3.1. Oversampling Techniques

Oversampling techniques consist of adding samples to the minority classes; in this study, two oversampling techniques were explored as described in the following:

- Adaptive Synthetic Sampling Approach (ADASYN) [31] creates samples in the minority classes according to their weighted density. The ADASYN allocates higher weights for instances that are difficult to classify using K-nearest neighbour (K-NN) classifier, where more synthetic samples are created for higher weights classes.
- Borderline Synthetic Minority Oversampling (BorderlineSMOTE) [32] identifies decision boundary (borderline) of minority samples and then synthetically generates samples in the minority class based on similarities in feature space along the identified borderline.

### 3.2. Undersampling Techniques

Undersampling techniques work by removing samples from the majority classes. In this study, two undersampling techniques were examined as described in the following:

- AllKNN [33] applies K-nearest neighbour (K-NN) classifier on majority class and removes all samples that have at least 1-nearest neighbour in the minority class, in order to make classes more separable
- Instance Hardness Threshold (IHT) [34] removes samples from majority classes with high probability of being misclassified

## 4. Hybrid Resampling (Combination of Over- and Undersampling)

The last category has investigated the hybrid approach that combines oversampling and undersampling techniques. This approach basically starts by oversampling minority classes followed by undersampling technique to remove majority classes samples that overlap minority classes samples. In this study, two hybrid techniques were examined as described in the following:

- Synthetic Minority Oversampling technique combined with edited nearest neighbour (SMOTEENN) [35] creates samples based on similarities in feature space, followed by edited nearest neighbour (ENN), which removes samples whose class label differs from the class of the majority of their K-nearest neighbours. In this study, 3-nearest neighbour algorithms with ENN are applied.
- Synthetic Minority Oversampling technique combined with Tomek link (SMOTETomek) [36] increases the number of minority class instances synthetically, similar to SMOTEENN, followed by Tomek link, which removes Tomek's link samples, which are pairs samples that belong to different classes and are each other's 1-nearest neighbours.

### 4.1. Classification and Hyperparameter Optimisation

Six different classifiers have been considered for classification: Artificial Neural Network based on Multilayer Perceptron (ANN-MLP) [37], Random Forest (RF) [38], support vector machine (SVM) [39], decision tree (DT) [40], logistic regression (LR) [41], and K-nearest neighbours (KNN) [42].

The six classifiers hyperparameters have been optimised using the Bayesian optimization algorithm [43, 44]. The Bayesian optimization algorithm utilises previous evaluations to predict the next set of hyperparameters that are close to the optimum. Consequently, reducing the number of evaluations requires achieving the best score. In this study, Bayes search method from scikit-optimize [45] has been used with 32 iterations and cross-validation.  Table 3 shows hyperparameters search spaces that have explored in this study.

### 4.2. Performance Metrics

Accuracy, precision, sensitivity, and specificity are the most commonly used metrics of classification algorithms performance [46], but such metrics are inadequate to assess classifiers as they are sensitive to data distribution [47]. Thus, metrics such as F1-score and geometric mean (G-mean) are frequently used for evaluating classifiers to balance between sensitivity and precision [17]. However, despite the fact that G-mean and F1-score decrease the effect classes distribution, they do not take into consideration the true negatives and classes contribution to overall performance [48]. Therefore, in addition to these metrics, advanced metrics such as Index of Balanced Accuracy (IBA) [48] and Area under the Curve (AUC) [49] have been used in this study in order to find an optimal system that does not bias to specific classes and does not rely on one metric:

(2) $$\begin{array}{c} \text{accuracy}=\frac{\text{TP}+\text{TN}}{\text{TP}+\text{TN}+\text{FP}+\text{FN}},\\ \text{precision}=\frac{\text{TP}}{\text{TP}+\text{FP}},\\ \text{sensitivity}=\text{TPR}=\frac{\text{TP}}{\text{TP}+\text{FN}},\\ \text{specificity}=\text{TNR}=\frac{\text{TN}}{\text{TN}+\text{FP}},\\ \text{F}1-\text{score}=\frac{2*\text{precision}*\text{sensitivity}}{\text{precision}+\text{sensitivity}},\\ G-\text{mean}=\sqrt{\text{sensitivity}\times \text{specificity}},\\ {\text{IBA}}_{\alpha }=\left(1+\alpha \cdot \left(\text{TPR}-\text{TNR}\right)\right)\cdot G{\text{Mean}}^{2}, \end{array}$$

where 0 ≤ *α* ≤ 1. TP, FP, TN, FN, TPR, TNR, and *α* refer, respectively, to true positive, false positive, true negative, false negative, true positive rate, true negative rate, and weighting factor.

## 5. Recommended Tasks Framework

A key aspect of a recommended system is to identify the best tasks or activities performed by PD patients to detect tremor severity. Therefore, a recommended tasks framework is proposed, as shown in Algorithm 1. The algorithm basically utilise classification performance metrics of different classifiers with and without resampling of different tasks from different datasets to identify best tasks.

After classification, the performance metrics of all datasets were collected separately. After that, the following steps were performed for each collected metric results independently. The highest value of each metric of each task has been identified in two cases, the first case when the dataset was classified without resampling and the second case with resampling. Then, an above-average rule has been applied for each dataset, where the values above average among all tasks have been selected. After that, the number of values above average counted for each task among all datasets.

In the final stage, the total number of all counters for all metrics for each task in all datasets was calculated and sorted in the descending order list. The list of tasks is grouped into three groups: recommended, neutral, and not recommended. Each group will contain six tasks from the datasets that have been performed during data collection.

### 5.1. Recommended Classifiers and Resampling Techniques Framework

After identifying the recommended tasks in the previous section, the results are used to identify the recommended classifier(s) and resampling technique(s).  Figure 3 presents the proposed framework to identify which classifiers, hyperparameters, and resampling techniques that achieved the highest accuracy for each task, and this will produce potential recommended systems that will be evaluated later in the following section (Potential Recommended Systems Evaluation).

The first stage is to highlight the classifier(s) and hyperparameters that achieved the highest accuracy with all resampling techniques, then selecting the most frequent classifier(s) that achieved the highest score. The second stage is to select resampling technique(s) with the highest count with selected classifier(s) in the first stage. If classifiers and resampling techniques were selected more than once in the previous stage, the third stage was applied to filter the results based on the highest validation score and then based on lowest fit time. The potential recommended systems saved for evaluation, which will be explained in the following section.

### 5.2. Potential Recommended Systems Evaluation

A number of saved potential recommended systems will be evaluated to determine the ideal system for deployment. The evaluation process utilised 15% of all datasets combined. The recommended system should estimate tremor severity regardless of used data in this study and should work well if the data is collected using the same sensors while subjects are performing the recommended tasks found in this study. Evaluation data was split into two parts, 10% was evaluated through the metrics as described in Performance Metrics section using the saved potential systems, and 5% was split into 20 samples used as external test data to be predicted as patient data.

The results of the first part of evaluation data, the 10%, were utilised to select top performance models (ideal models), and then the ideal models were tested and validated to predict the 5% external test data. The 5% test data was split into 20 separate samples to predict every sample overall tremor severity by calculating the value at which the probability mass function is the maximum.

## 6. Results and Discussions

The section is presented in three parts. The first part will discuss the recommended tasks. The recommended classifiers and resampling techniques are presented in the second part. The third part presents the potential recommended systems and final recommended system.

### 6.1. Recommended Tasks

Table 4 shows the results of one metric (accuracy) utilised to identify recommended tasks with resampling and without resampling, the highlighted values are above average among each dataset, while the count above average column shows values that are above average for datasets for each task. Closer inspection of the table shows that resampling techniques improved the accuracy significantly. However, classification accuracy off datasets follows the same trend when they resampled and when they did not resample. The same process has been applied for all metrics (AUC, F1-score, G-mean, and IBA).

Table 5 presents the results of above-average count of all metrics and groups the 18 tasks performed during data collection into three groups: recommended, neutral, and not recommended. It can be observed that tasks involving direct wrist movements have the lowest count (not recommended tasks), while tasks not involving direct wrist movements have the highest count (recommended tasks). The neutral tasks have count less than the recommended task but higher than not recommended tasks. A likely explanation is that these tasks do not involve direct wrist movements similar to not recommended task. So, another possible area of future research would be to investigate these tasks in more detail with different patients.

Together, these results provide important insights into tasks performed during data collection influence classification performance; therefore, this study presents recommended tasks (stairs down, sitting, stairs up, walking straight, walking while counting, and sit to stand) to be performed to measure tremor through wearable devices.

### 6.2. Recommended Classifiers and Resampling Techniques

The recommended classifier(s) and resampling technique(s) were identified following the framework, which was described in Recommended Classifiers and Resampling Techniques Framework section.  Figure 4 shows the results of first recommended task (strsd). In the first stage, two classifiers (ANN-MLP and SVM) have the highest count. In the second stage, three resampling techniques (ADASYN, BorderlineSMOT and SMOTETomek) have the highest count with both filtered classifiers in the first stage. In the next stage, SVM achieved the highest validation score 100%. Finally, based on fit time, SVM combined with ADASYN was found to be the best model to classify tremor of strsd task, which is the first potential recommended system. The same procedure applied for all recommended tasks to produce six potential systems is presented in Table 6. What is interesting about the data in this table is that all potential recommended systems include SVM as a classifier. In addition, the most common kernel is “rbf,” except system 4.

These findings suggest that SVM with oversampling and hybrid resampling techniques (ADASYN, BorderlineSMOTE, SMOTETomek, and SMOTEENN) performance is better than other classifiers and resampling techniques that have been examined in this study. However, in order to identify a recommended system, the potential systems were evaluated as discussed in Potential Recommended Systems Evaluation section. The performance of potential systems on the evaluation data (15%) is presented in Table 7. It is apparent from this table that system 6 achieved the highest performance with 98% accuracy, 98% F1-score, 98% G-mean, 97% IBA, and 100% AUC, while systems 4 and 5 achieved worst performance. Systems 1, 2, and 3 performance is lower than system 6 but better than others. Therefore, top 4 systems were evaluated through tremor severity prediction approach utilising the 5% (20 samples) external test data.  Table 8 shows the predictions results of all 20 samples of the top 4 systems. Systems 2 and 4 predicted all samples correctly, while systems 1 and 3 misclassified sample 19. System one was not able to classify sample 19 exactly as it gives the same probability for severities 3 and 0, while the actual severity is 3. On the other hand, system 3 classified the same sample as 0. Hence, this study suggests system 6 is a recommended system, since it performed better on evaluation and test data and the second choice is system 2 and then systems 1 and 3, respectively. The confusion matrix and Receiver Operating Characteristic (ROC) curve of the recommended system (System 6) are presented in Figures 5(a) and 5(b), respectively.

## 7. Study Limitations

We acknowledge that this study has a number of limitations. First, the sample size is small and may not be fully representative of the wider PD population. Second, the dataset was collected in one environment. Hence, results may differ if the environment is changed. Third, the recommended systems should be evaluated with different dataset that is collected independently of the used dataset and should be evaluated by different researchers to validate inter- and intrareliability.

## 8. Conclusion and Future Work

The main goal of the current study was to identify task-oriented intelligent solution that can be used to measure tremor severity using wearable devices combined with machine learning techniques. This study has been one of the first attempts to thoroughly examine the influence of tasks performed during data collection on classification performance. Furthermore, a comprehensive approach was used to identify best classifiers, classifiers hyperparameters, and resampling techniques in combination with signal processing and robust features extraction techniques. Different metrics, including accuracy, F1-score, G-mean, IBA, and AUC, have been used to identify the recommended system using a novel algorithm to avoid bias. In general, ADL tasks that involve direct wrist movements are not suitable for tremor severity assessment such as drawing, writing, drinking, folding a towel, typing, organizing sheets in a folder, and assembling nuts and bolts. On the other hand, tasks that do not involve direct wrist movements achieved high performance of tremor severity classification. In addition, resampling techniques can improve classification performance. In this study, the recommended system has been suggested to evaluate tremor severity from data that was collected using two types of wearable devices, while patients are either on medication or off medication. The recommended system consists of three main components, which are classifier, resampling technique, and the tasks to be performed during data collection. The findings of this study suggest that the best system is the SVM classifier combined with BorderlineSMOTE oversampling technique, and the tasks are sitting, stairs up and down, walking straight, walking while counting, and standing. The suggested recommended system has been tested using evaluation data from two wearable devices and achieved 98% accuracy, 98% F1-score, 97% IBA, 98% G-mean, and 99% AUC. In addition, it has been tested to predict tremor severity of test data from both wearable devices, and it was able to predict all samples correctly.

For future studies, it is suggested to test the recommended system with different datasets and also to explore more ADL tasks and different wearable devices in different environments, including free-living tasks at home.

## Figures and Tables

**Figure 1:** Proposed framework for tremor severity classification.

**Figure 2:** Tremor datasets.

**Figure 3:** Recommended classifiers and resampling techniques.

**Figure 4:** Recommended classifiers and resampling techniques results (strsd).

**Figure 5:** Recommended system (system 6) confusion matrix and ROC curve.

**Algorithm 1:** Recommended tasks algorithm.

**Table 1:** Imbalanced classes (severities) distribution.

Tremor severity	GENEActiv		Pebble		Total
(Class)	Day 1	Day 4	Day 1	Day 4	(*n*=103080)
0	18843	16860	19389	17215	72307
1	5845	6534	4491	4421	21291
2	2185	2921	1357	1112	7575
3	845	676	117	103	1741
4	43	53	11	59	166

**Table 2:** Extracted features and their descriptions.

Feature	Domain	Formula
Above mean	T and F	|*W*^+^| : *W*^+^={*a*_*t*_ ∈ *W* : *a*_*t*_ > (1/*W*_*l*_∑_*t*=0_^*W*_*t*_^*a*_*t*_)}
Below mean	T and F	|*W*^−^| : *W*^−^={*a*_*t*_ ∈ *W* : *a*_*t*_ < (1/*W*_*l*_∑_*t*=0_^*W*_*t*_^*a*_*t*_)}
Autocorrelation	T and F	$1/\left(W_{l}-l\right)s_{w}^{2}\sum_{t=0}^{W_{l}-l}\left(a_{t}-\bar{a}\right)\left(a_{t+l}-{\bar{a}}_{w}\right)$
Complexity-invariant distance (CID)	T and F	$\sqrt{\sum_{t=1}^{W_{l}-1}{\left(a_{t}-a_{t+1}\right)}^{2}}$
Sample entropy	T and F	log_*e*_(*A*^*m*+1^(*r*)/*A*^*m*^(*r*))
Kurtosis	T and F	$1/W_{l}\sum_{t=0}^{W_{l}}{\left(a_{t}-{\bar{a}}_{w}\right)}^{4}/s_{w}^{4}$
Skewness	T and F	$1/W_{l}\sum_{t=0}^{W_{l}}{\left(a_{t}-{\bar{a}}_{w}\right)}^{3}/s_{w}^{3}$
Standard deviation	T and F	$\sqrt{\sum_{t=0}^{W_{l}}{\left(a_{t}-{\bar{a}}_{w}\right)}^{2}/W_{l}-1}$
Max	T and F	$\underset{t=0}{\overset{W_{l}}{\max}}a_{t}$
Mean	T and F	1/*w*∑_*t*=0_^*W*_*l*_^*a*_*t*_
Median	T and F	$\left\{\begin{array}{cc} a_{t}^{\left(i\right)} & :i=\left(W_{l}^{\left(𝒪\right)}+1\right)/2\\ \left(a_{t}^{\left(i\right)}+a_{t}^{\left(i+1\right)}\right)/2 & :i=W_{l}^{\left(ℰ\right)}/2 \end{array}\right.$
Sum of absolute differences (SAD)	T and F	∑_*l*=0_^*W*_*i*_^|*a*_(*t*+1)_ − *a*_*t*_|
Energy	T and F	∑_*t*=0_^*W*_*l*_^*a*_*t*_^2^
Peaks	T	|*P*| : *P*={max{*a*_(*n*+*m*+*k*)_}_*k*=−*n*_^*n*^}_*m*=0_^*W*_*l*_−(2*n* − 1)^
Amplitude of peak PSD	F	$\max_{W}\left(\sqrt{\text{PSD}}\right)=\max_{a_{t}\in W}\left(\sqrt{1/W\left|\sum_{t=0}^{W_{l}-1}a_{t}e^{{\left(-j2\pi kt/W_{l}\right)}_{2}}\right|}\right)$
Median frequency	F	*f*_med_ : (∑_*f*=*f*_*t*__^*f*_med_^PSD)=(∑_*f*=*f*_med__^*f*_med_^PSD)=(1/2(∑_*f*=*f*_*t*__^*f*_h_^PSD))
Frequency dispersion	F	*f*_disp_=2*f*_step_ : (∑_*f*_med_+*f*_step__^*f*_med_+*f*_step_^PSD=68/100∑_*f*=*f*_*t*__^*f*_*h*_^PSD)
Fundamental frequency	F	$f_{\text{fund}}:{\text{PSD}}_{\text{fund}}=\underset{f_{l}}{\overset{f_{h}}{\max}}\left\{\text{PSD}\right\}$
Frequency difference	F	*f*_med_ − *f*_fund_
Spectral centroid amplitude (SCA)	F	∑_*f*=*f*_*l*__^*f*_*h*_^(*f*)(PSD)/∑_*f*=*f*_^*f*_*h*_^(*f*)
Maximum weighted PSD	F	$\underset{f_{l}}{\overset{f_{h}}{\max}}\left\{\left(f\right)\left(\text{PSD}\right)\right\}$

*W*^+^: window subset contains elements above the mean; *W*^−^: window subset contains elements below the mean; *W*_*l*_: window length (number of samples); *a*_*t*_: the acceleration at time *t*; *l*: the lag. ${\bar{a}}_{w}$: window's samples mean; *s*_*w*_: window's samples standard deviation; *A*^*m*^(*r*): the probability that two vectors of *m* points within a one window would match; *A*^*m*+1^(*r*): the probability that two vectors of *m*+1 points within one window would match; *W*_*l*_^(*𝒪*)^: window length is odd; *W*_*l*_^(*ℰ*)^: window length is even; *i*: an element position (index) in the window {*W*}; *n*: number of neighbours; *a*_(*n*+*m*+*k*)_: the acceleration at a time (*n*+*m*+*k*); *W*: the selected window; *e*^−*j*2*π*/*W*_*l*_^: the primitive *N*th root of unity; *f*_dis_: the dispersion frequency in the selected window; *f*: frequency bin; *f*_*l*_: the lowest frequency in the selected window; *f*_*h*_: the highest frequency in the selected window; *f*_step_: the range between the median frequency and the lower bound of dispersion frequency, which is equal to the range between median frequency and the higher bound of dispersion frequency, that is, 2*f*step is the range between lower and higher bound of of dispersion frequency; PSD_fund_: the PSD at fundamental frequency.

**Table 3:** Classifiers' hyperparameters search spaces.

Classifier	Hyperparameters search spaces
ANN-MLP	batch_size: [32, 64, 512]
	Epochs: [200, 300]
	Neurons: Integer (60, 100)
	Optimizer: [SGD, RMSprop, Adam, Adadelta, Adagrad, Adamax, Nadam]
	Activation: [relu, tanh, selu, elu, exponential]

KNN	n_neighbors: Integer (1, 20)
	Weights: [Distance, uniform]
	Algorithm: [Brute, ball_tree, kd_tree]
	Metric: [Minkowski, euclidean, manhattan]
	leaf_size: Integer (1, 20)
	*p*: Integer(1, 2)

RF	n_estimators: Integer(10, 250)
	max_features: Integer(1, 102)
	max_depth: Integer(5, 100)
	min_samples_split: Integer(2, 20)
	min_samples_leaf: Integer(1, 20)
	Criterion: [gini, entropy]

DT	max_features: Integer(1, 102)
	max_depth: Integer(5, 100)
	min_samples_split: Integer(2, 20)
	min_samples_leaf: Integer(1, 20)
	Criterion: [gini, entropy]

LR	Penalty: [l2, none]
	C: [1*e* − 2, 1*e* − 1, 1*e*0, 1*e*1]
	Solver: [Newton-cg, lbfgs, sag, saga]
	max_iter: Integer(1, 1000)

SVM	C: [1, 2, 3, 4, 5, 6, 7, 8, 9, 10]
	Gamma: [0.1, 0.01, 0.001]
	Degree: (1, 5)
	Kernel: [Linear, poly, rbf, sigmoid]

**Table 4:** Task highest accuracy of all classifiers and values above average counts.

	Accuracy								
	Without resampling				With resampling				Count above average
	G-1 (%)	G-4 (%)	P-1 (%)	P-4 (%)	G-1 (%)	G-4 (%)	P-1 (%)	P-4 (%)	
drawg	66	55	88	95	93	91	95	99	3
drnkg	66	58	72	79	93	93	96	97	0
fldng	71	63	75	80	94	91	95	96	0
ftnl	77	76	65	62	97	96	95	96	3
ftnr	53	68	76	86	90	98	97	99	3
ntblt	71	63	71	75	95	94	95	96	0
orgpa	66	75	67	77	96	98	96	97	2
raml	77	79	68	59	96	97	98	94	4
ramr	68	59	82	85	96	91	98	99	4
typng	77	71	75	67	96	93	97	96	1
sittg	78	75	87	93	100	98	98	99	8
stndg	72	65	77	76	100	98	99	97	3
strsd	94	81	89	90	100	100	100	100	8
strsu	80	86	90	100	100	100	100	100	8
ststd	86	79	88	81	100	99	99	100	7
wlkgc	76	74	90	83	98	96	99	98	7
wlkgp	72	73	88	84	96	97	98	98	6
wlkgs	80	79	90	88	99	98	100	99	8
Average	74	71	80	81	97	96	98	98	

G-1: GENEActiv-Day 1; G-4: GENEActiv-Day 4; P-1: Pebble-Day 1; P-4: Pebble-Day 4.

**Table 5:** Tasks of above-average count for all metrics.

	Task	Count above average					
		Accuracy	AUC	F1-score	*G*-mean	IBA	Total
Recommended tasks	strsd	8	8	8	8	8	40
	sittg	8	7	8	8	8	39
	strsu	8	8	8	6	6	36
	wlkgs	8	8	8	6	6	36
	wlkgc	7	8	7	5	5	32
	ststd	7	7	7	5	4	30

Neutral tasks	ftnr	3	6	4	6	5	24
	raml	4	6	3	6	5	24
	wlkgp	6	7	6	2	3	24
	ramr	4	5	4	5	5	23
	stndg	3	7	3	5	5	23
	ftnl	3	4	3	4	4	18

Not recommended task	orgpa	2	6	2	2	2	14
	drawg	3	2	3	2	2	12
	typng	1	5	1	1	1	9
	fldng	0	4	0	2	2	8
	drnkg	0	3	0	1	1	5
	ntblt	0	1	0	0	0	1

**Table 6:** Potential recommended systems.

System	Task	Classifier	Resample technique	Validation score (%)	Hyperparameters	Mean fit time
System 1	strsd	SVM	ADASYN	100.00	*C*=10, degree=1, gamma=0.1, kernel=*rbf*	2.549183011
System 2	sittg	SVM	ADASYN	99.47	*C*=6, degree=5, gamma=0.1, kernel=*rbf*	5.469041586
System 3	wlkgs	SVM	ADASYN	98.34	*C*=10, degree=4, gamma=0.1, kernel=*rbf*	4.719249964
System 4	strsu	SVM	SMOTETomek	100.00	*C*=1, degree=5, gamma=0.001, kernel=linear	0.045000315
System 5	wlkgc	SVM	SMOTEENN	98.46	*C*=10, degree=1, gamma=0.1, kernel=*rbf*	1.642106652
System 6	ststd	SVM	BorderlineSMOTE	99.14	*C*=3, degree=5, gamma=0.1, kernel=*rbf*	6.840166569

**Table 7:** Potential systems performance.

System	Classifier	Resample technique	Accuracy (%)	*F*1-score (%)	IBA (%)	*G*-mean (%)	AUC (%)
System 1	SVM	ADASYN	97	97	96	98	99
System 2	SVM	ADASYN	97	97	96	98	99
System 3	SVM	ADASYN	97	97	96	98	100
System 4	SVM	SMOTETomek	96	96	94	97	99
System 5	SVM	SMOTEENN	93	93	90	95	99
System 6	SVM	BorderlineSMOTE	98	98	97	98	100

**Table 8:** Top four systems tremor severity predictions.

Sample data	Actual severity	Predicted severity			
		System 1	System 2	System 3	System 6
Sample_01	0	0	0	0	0
Sample_02	1	1	1	1	1
Sample_03	2	2	2	2	2
Sample_04	3	3	3	3	3
Sample_05	4	4	4	4	4
Sample_06	0	0	0	0	0
Sample_07	1	1	1	1	1
Sample_08	2	2	2	2	2
Sample_09	3	3	3	3	3
Sample_10	4	4	4	4	4
Sample_11	0	0	0	0	0
Sample_12	1	1	1	1	1
Sample_13	2	2	2	2	2
Sample_14	3	3	3	3	3
Sample_15	4	4	4	4	4
Sample_16	0	0	0	0	0
Sample_17	1	1	1	1	1
Sample_18	2	2	2	2	2
Sample_19	3	**(3, 0)**	3	**(0)**	3
Sample_20	4	4	4	4	4

The misclassified samples are in bold.

## Data Availability

The MJFF Levodopa Response Trial data used to support the findings of this study are restricted by the Michael J. Fox Foundation in order to protect the privacy of study participants. Data are available from Michael J. Fox Foundation datasets (https://www.michaeljfox.org/news/levodopa-response-study) for researchers who meet the criteria for access to confidential data.
